# Evaluation of Daily CT for EPID-Based Transit *In Vivo* Dosimetry

**DOI:** 10.3389/fonc.2021.782263

**Published:** 2021-11-02

**Authors:** Bin Feng, Lei Yu, Enwei Mo, Liyuan Chen, Jun Zhao, Jiazhou Wang, Weigang Hu

**Affiliations:** ^1^ Department of Radiation Oncology, Fudan University Shanghai Cancer Center, Shanghai, China; ^2^ Department of Oncology, Shanghai Medical College, Fudan University, Shanghai, China; ^3^ Shanghai Key Laboratory of Radiation Oncology, Shanghai, China

**Keywords:** portal dosimetry, EPID, quality assurance, IMRT verification, Monte Carlo method

## Abstract

**Purpose:**

The difference in anatomical structure and positioning between planning and treatment may lead to bias in electronic portal image device (EPID)-based *in vivo* dosimetry calculations. The purpose of this study was to use daily CT instead of planning CT as a reference for EPID-based *in vivo* dosimetry calculations and to analyze the necessity of using daily CT for EPID-based *in vivo* dosimetry calculations in terms of patient quality assurance.

**Materials and Methods:**

Twenty patients were enrolled in this study. The study design included eight different sites (the cervical, nasopharyngeal, and oral cavities, rectum, prostate, bladder, lung, and esophagus). All treatments were delivered with a CT-linac 506c (UIH, Shanghai) using 6 MV photon beams. This machine is equipped with diagnosis-level fan-beam CT and an amorphous silicon EPID XRD1642 (Varex Imaging Corporation, UT, USA). A Monte Carlo algorithm was developed to calculate the transmit EPID image. A pretreatment measurement was performed to assess system accuracy by delivering based on a homogeneous phantom (RW3 slab, PTW, Freiburg). During treatment, each patient underwent CT scanning before delivery either once or twice for a total of 268 fractions obtained daily CT images. Patients may have had a position correction that followed our image-guided radiation therapy (IGRT) procedure. Meanwhile, transmit EPID images were acquired for each field during delivery. After treatment, all patient CTs were reviewed to ensure that there was no large anatomical change between planning and treatment. The reference of transmit EPID images was calculated based on both planning and daily CTs, and the IGRT correction was corrected for the EPID calculation. The gamma passing rate (3 mm 3%, 2 mm 3%, and 2 mm 2%) was calculated and compared between the planning CT and daily CT. Mechanical errors [ ± 1 mm, ± 2 mm, ± 5 mm multileaf collimator (MLC) systematic shift and 3%, 5% monitor unit (MU) scaling] were also introduced in this study for comparing detectability between both types of CT.

**Result:**

The average (standard deviation) gamma passing rate (3 mm 3%, 2 mm 3%, and 2 mm 2%) in the RW3 slab phantom was 99.6% ± 1.0%, 98.9% ± 2.1%, and 97.2% ± 3.9%. For patient measurement, the average (standard deviation) gamma passing rates were 87.8% ± 14.0%, 82.2% ± 16.9%, and 74.2% ± 18.9% for using planning CTs as reference and 93.6% ± 8.2%, 89.7% ± 11.0%, and 82.8% ± 14.7% for using daily CTs as reference. There were significant differences between the planning CT and daily CT results. All p-values (Mann–Whitney test) were less than 0.001. In terms of error simulation, nonparametric test shows that there were significant differences between practical daily results and error simulation results (p < 0.001). The receiver operating characteristic (ROC) analysis indicated that the detectability of mechanical delivery error using daily CT was better than that of planning CT. AUC_Daily CT_ = 0.63–0.96 and AUC_Planning CT_ = 0.49–0.93 in MLC systematic shift and AUC_Daily CT_ = 0.56–0.82 and AUC_Planning CT_ = 0.45–0.73 in MU scaling.

**Conclusion:**

This study shows the feasibility and effectiveness of using two-dimensional (2D) EPID portal image and daily CT-based *in vivo* dosimetry for intensity-modulated radiation therapy (IMRT) verification during treatment. The daily CT-based *in vivo* dosimetry has better sensitivity and specificity to identify the variation of IMRT in MLC-related and dose-related errors than planning CT-based.

## Introduction

An electronic portal image device (EPID) is a useful tool in radiotherapy. These devices were initially developed to improve the accuracy of patient setup (1) in the 1980s and have become important equipment for quality control (QC) and quality assurance (QA) in radiotherapy. By obtaining MV-level transmission images through a fluorescence imaging system, an EPID can be used for light field consistency verification, isocenter verification, treatment bed movement accuracy verification, multileaf collimator (MLC) QC, and pretreatment patient-specific QA (2–8).

For pretreatment patient-specific QA, compared to ionization chambers, films, and two-dimensional (2D) matrices, EPID-based measurements, such as portal dosimetrics (Varian, Palo Alto, CA, USA), have advantages in easy acquisition, low cost, and fast analysis (9).

In addition, EPID-based *in vivo* dosimetrics, which measure transmission images during patient delivery for intensity-modulated radiation therapy (IMRT) and volumetric modulated arc therapy (VMAT), have been demonstrated to be feasible in recent years (10–12). Fuangrod et al. (13) used statistical process control and other methods to compare the consistency of the calculated and actually measured dose accumulation points in real time, and the dose delivery error could be found within 2 s. Miri et al. (14) used Varian’s aS1200 DMI panel to develop a QA model for IMRT delivery verification. In addition, Willett et al. (15) tested this device for routine FFF QA and dosimetry measurement. Chuter et al. (16) used the Swedish Elekta iViewGT for dose verification, and their results were consistent with the verification results of the 3D dose-verification system Delta4 (ScandiDos, Sweden). Spreeuw et al. (17) used an independent algorithm to calculate EPID portal images to reconstruct the 3D dose distribution, and the dose delivery error could be detected at 5–10 s.

However, these studies were all calculated based on the phantom or planning CT (pCT). The disadvantage of pCT is that it is difficult to distinguish what caused the drop in the gamma pass rate. To solve this problem, a few studies were focused on daily CT (dCT) images.

Olaciregui-Ruiz et al. (18) converted the reference pCT image into a synthetic dCT image. The patient’s setup position and changes in the patient’s anatomy are simulated to evaluate the sensitivity of 3D EPID transmission dose measurement (19).

The synthetic image is not an ideal solution for transmission image calculation, as it may not represent the real patient’s anatomy during treatment. **Figure 1** illustrates two examples of actual treatment variations between pCT and dCT. In practice, the patient’s internal organs do not simply expand or contract as seen in prior synthetic dCT research (18). Furthermore, previous study showed that first fraction is most effective for EPID-based dosimetry verification (20). Therefore, pCT may not be appropriate as a reference image for *in vivo* dosimetry during clinical practice.

**Figure 1:** Anatomical variations between planning CT (pCT) and daily CT (dCT). **(A)** pCT of a rectal patient; **(B)** dCT of a rectal patient; **(C)** pCT of an NPC patient; and **(D)** dCT of an NPC patient. NPC, Nasopharyngeal Carcinoma.

Reference imaging is one of the key concerns in EPID transmission studies. Both previously mentioned strategies (pCT and synthetic dCT) cannot fully reflect anatomical changes. Moreover, because of the lack of CT of the patient at the time of delivery, the impact of using pCT as a reference has not been fully investigated (18, 19).

Recently, a new type of linac (CT-linac 506c, United Image Healthcare, Shanghai, China) was developed and used in the clinic. It can obtain diagnosis-level CT images before treatment delivery and acquire transmission EPID images during treatment. This device provides the feasibility of using the real dCT as a reference for EPID-based *in vivo* dosimetry system development.

In this study, we used dCT instead of pCT as a reference for EPID-based *in vivo* dosimetry calculations and investigated the detectability of using dCT on EPID-based *in vivo* dosimetry calculations in terms of patient QA. We used actual patient treatment data to assess machine-related error detectability between dCT and pCT. Meanwhile, we try to find the threshold for error detection.

## Materials and Methods

### Study Design

**Figure 2** shows the whole study design. This study can be divided into two parts: pretreatment QA and *in vivo* dosimetry. Twenty patients with different tumor sites were enrolled in this study. A pretreatment QA was performed to assess algorithm accuracy. During treatment, patients may receive CT scanning before delivery according to our clinical protocol. Patients may have position correction by this dCT. A transmission EPID image was acquired during patient delivery. After treatment, dCT and pCT information was collected for data analysis.

**Figure 2:** The study workflow.

### Linear Accelerator, Electronic Portal Image Device, and Fan-Beam CT

All deliveries and measurements were performed on a UIH CT-Linac 506c (**Figure 3**), which was developed by the United Imaging Company (Shanghai, China). This device has been integrated with diagnosis-level fan-beam CT (FBCT), which can scan the patient directly before treatment. It has one photon energy (6 MV) and 80 pairs of MLCs (0.5-mm width). Both static IMRT (sIMRT) and dynamic IMRT (dIMRT) are supported by this device.

**Figure 3:** The CT-Linac 506c.

The UIH CT-linac 506c is equipped with a Varex Imaging XRD 1642 amorphous silicon EPID. The EPID has a 40.96 × 40.96-cm^2^ detector effective area that contains 1,024 × 1,024 pixels with a 0.4-mm pixel size in 1 × 1 binning mode or 512 × 512 pixels with a 0.8-mm pitch in 2 × 2 binning mode. The maximum frame rate reaches 15 frames per second (fps) in 1 × 1 binning mode or 30 fps in 2 × 2 binning mode. The source-to-image distance (SID) is 145 cm; thus, the spatial resolution in the ISO plane is ~0.27 mm (1 × 1 binning) or ~0.55 mm (2 × 2 binning).

The diagnosis-level FBCT was equipped on the back of this accelerator, as shown in **Figure 3**. Three image scanning protocols were used in this study, namely, head and neck, chest, and pelvic. The imaging doses were 51.2, 8.6, and 13.4 mGy for head and neck, chest, and pelvic tissue, respectively. The 10% modulation transfer functions (MTF 10%) were 8.2 ± 0.1 lp/cm, 5.1 ± 0.2 lp/cm, and 5.2 ± 0.1 lp/cm for the head and neck, chest, and pelvic areas, respectively. The image uniformity was 0.5% in the head and neck and 0.2% in both the chest and pelvis.

### Patients and Plans

Twenty patients with different tumor sites were enrolled in this study. All treatment plans were developed by physicists with 5–10 years of experience. These plans were clinically approved and used for patient treatment. All plans use the IMRT technique. Two IMRT delivery methods were used, including sIMRT and dIMRT.

### Pretreatment Quality Assurance

All plan parameters, including monitor units (MUs), gantry, collimator, couch angles, jaws, and MLC leaf position, were copied from the original plan (21). This QA plan would then be executed on an RW3 slab phantom (PTW, Freiburg, Germany; **Figure 4**). In this study, 15 pieces of 10-mm-thick plates were used (**Figure 4**).

**Figure 4:** The quality assurance (QA) phantom, the RW3 slab phantom (PTW, Freiburg).

The reference EPID transmission images were calculated by the Monte Carlo algorithm (22–24). In the calculation, the setting for the total particle number was 3.0 × 10^9^, and the uncertainty was 0.01 (25).

After the QA plan delivery, the EPID transmission was acquired and gray corrected. Gamma analysis was used for evaluation.

### Patient Delivery

Patients received online CT scanning before delivery either once or twice during the whole treatment course. Details on the CT scanning information for each patient are presented in **Table 1**. This image was used for patient position correction by rigid image registration. Patients may have had position correction before delivery when they had a more than 3-mm shift according to our clinical protocol. EPID transmission images were collected each time, even when no CT scanning is performed.

**Table 1:** Patient cohort characteristics.

	Disease site	Beam number	Number of fractions	Prescription dose/cGy	Technology	Daily CT number
Patient 1	Prostate	7	25	4,500	sIMRT	2
Patient 2	Nasopharyngeal	6	30	6,000	sIMRT	2
Patient 3	Cervical	7	25	5,000	sIMRT	2
Patient 4	Rectum	7	25	5,000	sIMRT	2
Patient 5	Esophagus	9	34	6,120	dIMRT	2
Patient 6	Oral cavity	9	33	6,600	dIMRT	1
Patient 7	Rectum	7	25	5,000	sIMRT	2
Patient 8	Rectum	7	25	5,000	sIMRT	2
Patient 9	Oral cavity	9	30	6,000	dIMRT	2
Patient 10	Rectum	7	25	5,000	sIMRT	2
Patient 11	Rectum	7	25	5,000	sIMRT	2
Patient 12	Rectum	7	25	5,000	sIMRT	2
Patient 13	Rectum	7	25	5,000	sIMRT	2
Patient 14	Lung	6	28	5,040	dIMRT	2
Patient 15	Parotid gland	6	30	6,600	dIMRT	2
Patient 16	Parotid gland	6	30	6,000	dIMRT	2
Patient 17	Rectum	7	25	5,000	sIMRT	2
Patient 18	Rectum	7	25	5,000	sIMRT	2
Patient 19	Rectum	7	25	5,000	sIMRT	2
Patient 20	Rectum	7	25	5,100	sIMRT	1

dIMRT, dynamic intensity-modulated radiation therapy; sIMRT, static intensity-modulated radiation therapy.

### Transmission Image Calculation

We used the Monte Carlo algorithm for transmission image calculation. Briefly, phase space files of photons and electrons were used to generate scoring plane images at the EPID position. Then, the detector response and lateral scatter were applied on this image. This total response can be transferred to a grayscale image by dose/MU grayscale calibration.

For each patient, pCT-based transmission images were calculated for each fraction. Patients may have had 25~35 pCT-based transmission images for each field, which depended on the number of treatment fractions. However, the patients only received 1~2 dCT scans during the whole treatment course. For appropriate comparison, only fractions with dCT were selected for analysis. In addition, both images consider the setup shift as we mention below.

Patients can have a setup shift between planning and delivery. Thus, directly using the pCT isocenter for dCT-based transmission image calculations may not be appropriate. To reflect the actual setup position during delivery and to remove the influence of setup error, we moved the isocenter of pCT for dCT-based transmission image calculation. This isocenter shift was acquired by 3D image rigid registration between the pCT and dCT. For patients who have an image-guided radiation therapy (IGRT) correction, the correction shift will be accounted for to obtain the patient’s real position during delivery.

For dCT-based transmission image calculation, we used a system-provided isocenter that already represents the actual delivery isocenter.

### Measured Image Correction

In previous studies, we have considered image calibration for panel and CT scans; FBCT was estimated by assessing the volume CT dose index (CTDI) for each protocol (26). Measured images were corrected before comparison. EPID is mounting at a frame that is supported by a mechanical arm. The mechanical arm is out of the field, so the backscatter could be ignored. The following corrections were performed:

- Geometry correction. Correction of the geometric displacement of the center of the light source beam relative to the center of the EPID flat panel detector during the rotation of the gantry angle. Due to the effect of gravity, the distance from source to detector and the relative position of the imager need a little correction that is based on a calibration method that stems from the imaging of 1.5 MV imaging beam line (IBL) from the beam-defining head (BDH) in every direction of gantry.
- Dead pixel correction. Correction of the value of abnormal or unresponsive pixel units in the image.
- Dark current correction. Additionally known as dark field correction, the electronic noise of the detector is corrected when there is no optical signal.
- Detector response correction. Additionally known as gain correction, the inconsistency of the signal response of the pixel unit of the detector is corrected.

### Image Analysis

Here, we used local Gamma analysis to compare the measured and calculated transmission EPID images (27). No 2D image registration was performed. Three criteria were used in the Gamma analysis. The dose difference and distance to agreement (DTA) for the gamma passing rate approach criteria were 3% 3 mm, 3% 2 mm, and 2% 2 mm, respectively. The Gamma analysis threshold was 10% (points below 10% of the maximum dose point were excluded).

### Statistical Method

Data obtained from the Gamma analysis were compared using a Mann–Whitney test. The criterion for significance for all analyses was set at P = 0.05.

To analyze the correlation between the results of dCT and pCT, the Pearson correlation coefficient was calculated.

### Simulation of Treatment Variability and Receiver Operating Characteristic Analysis

In order to separate machine-related and patient-related errors, the systematic shifting of all MLC positions and the dose bias were introduced in dCT-based treatment plan and predicted portal images, including the following:

- The MU were scaled by ±3%, ± 5%.
- All MLC positions were systematically shifted by ±1, ± 2, and ±5 mm.

In this study, we consider that dCT and IGRT technology maximally fixed the anatomy-related changes and setup error. Therefore, machine-related error can be separated and detected during treatment. When the gamma index is too low to accept, it prompts the physicist to check the machine.

The receiver operating characteristic (ROC) curves were used in this study for assessing the detectability of mechanical offsets. Treatment plan was divided into two groups: (1) unmodified dCT-based plan and (2) modified dCT-based plan. The ROC curves were plotted by varying gamma passing rate threshold.

## Results

### Pretreatment Quality Assurance

The gamma passing rates in pretreatment QA were 99.57% ± 1.09%, 98.91% ± 2.09%, and 97.12% ± 3.99% [the mean ± standard deviation (STD)] for the 3 mm 3%, 2 mm 3%, and 2 mm 2% criteria, respectively. With the 3 mm 3% criteria, all field pass rates were higher than 95%, and four fields were lower than 98%. For the 2 mm 3% criteria, one field did not pass 90%. With the 2 mm 2% criteria, there were five fields lower than 90%.

**Figure 5** shows an example of the pretreatment QA for patient 1, including the measured image and calculated image. **Figures 5C, D** show the gamma map (2 mm 2%) and profile for comparing the measurements and calculation.

**Figure 5:** The cases of pretreatment quality assurance (QA). **(A)** An electronic portal image device (EPID)-measured image. **(B)** A phantom model-based calculated image. **(C)** The corresponding Gamma analysis results. **(D)** Profiles representing inlines and crosslines are shown in panels **(A, B)**.

### Planning CT Results

The gamma passing rates by using pCT for reference transmission image calculation were 90.02% ± 11.52%, 85.17% ± 14.29%, and 77.70% ± 16.96% (the mean ± standard deviation) for the 3 mm 3%, 2 mm 3%, and 2 mm 2% criteria, respectively (the red tag in **Figure 6**).

**Figure 6:** The Gamma analysis results of planning CT (pCT) and daily CT (dCT). The red box diagram represents the pCT results. The blue box represents the dCT results.

### Daily CT Results

The gamma passing rates by using the dCT for reference transmission image calculation were 95.04% ± 6.45%, 92.12% ± 8.70%, and 86.84% ± 11.94% (the mean ± standard deviation) for the 3 mm 3%, 2 mm 3%, and 2 mm 2% criteria, respectively (the blue tag in **Figure 6**).

There was a significant difference between the pCT and dCT results. The mean ± standard deviation was 2.46 ± 3.31 (3 mm 3%), 3.79 ± 3.75 (2 mm 2%), and 5.43 ± 5.61 (2 mm 2%). The Mann–Whitney test results on the gamma passing rate between the dCT and pCT were p = 0.001 (3 mm 3%), p = 0.001 (2 mm 3%), and p = 0.001 (2 mm 2%).

**Figure 7** is the scatter plot of the dCT and pCT results. **Figures 7A–C** represent the comparison results under the criteria of 3 mm 3%, 2 mm 3%, and 2 mm 2%, respectively. Among 268 beams, 206 (76.87%), 212 (79.10%), and 204 (76.12%) beams had better performance with dCT. The Pearson correlation coefficients were 0.692 (3 mm 3%), 0.684 (2 mm 3%), and 0.656 (2 mm 3%).

**Figure 7:** Gamma analysis results of the daily CT-based *vs.* planning CT-based methods. The daily CT-based results indicate a higher gamma passing rate; **(A)** 3 mm 3%; **(B)** 2 mm 3%; and **(C)** 2 mm 2%.

The cases of EPID-based *in vivo* dosimetry during treatment is shown in **Figure 8**. Using the 3 mm 3% criterion, the gamma passing rates of prostate, rectum, nasopharyngeal, and lung were 98.19%, 85.89%, 98.46%, and 82.80%, respectively, as calculated by the pCT and 99.32%, 81.45%, 99.15%, and 89.31%, respectively, as calculated by the dCT.

**Figure 8:** The cases of electronic portal image device (EPID)-based *in vivo* dosimetry during treatment. **(A)** An EPID-measured image. **(B)** A planning CT (pCT)-based calculated image. **(C)** A daily CT (dCT)-based calculated image. **(D)** The corresponding Gamma analysis results between the pCT and measurement. **(E)** The corresponding Gamma analysis results between the dCT and measurement. **(F)** Profiles representing inlines and crosslines are shown in panels **(A–C)**.

### Error Analysis

For 20 patients who were delivered between May 2020 and June 2021, a summary of the gamma analysis for introducing each error is shown in **Table 2**. The gamma pass rate decreased by 9.9% (2 mm 2%) and 3.26% (3 mm 3%) on average when ±1 mm MLC deviation was introduced. In ±2 mm MLC shift, the average gamma passing rate was 60.64% at 2 mm 2% and 81.6% at 3 mm 3%. Furthermore, in ±5 mm MLC shift, the mean passing rate decreased to 42.66% at 2 mm 2%. Similarly, in 3% MU scaling, the gamma passing rate dropped 6.42% (2 mm 2%) and 2.66% (3 mm 3%). In 5% MU scaling, the mean gamma passing rate is 62.97% (2 mm 2%) and 84.64% (3 mm 3%). **Figure 9** shows the distribution of gamma passing rate for dCT-based plan and a plan with a mechanical error. The best threshold was found by finding a cutoff where true positive rate (TPR) is high and false positive rate (FPR) is low. For a given threshold, sensitivity and specificity can be calculated (**Figure 9**).

**Table 2:** Mean and standard deviation of gamma passing rate for different error introduction and best threshold in varying variations.

	Failure mode	dCT_error_ vs. measurement	dCT_error_ vs. measurement	Best threshold (2 mm 2%)
		2 mm 2% (γ_mean_% ± STD)	3 mm 3% (γ_mean_% ± STD)	
Gold criterion		82.8 ± 14.7	93.6 ± 8.2	–
MLC systematic shift	± 1 mm	72.90 ± 12.36	90.34 ± 10.31	76.80
	± 2 mm	60.64 ± 11.59	81.60 ± 11.19	76.88
	± 5 mm	42.66 ± 11.89	57.44 ± 12.61	66.25
MU scaling	3%	76.38 ± 14.94	90.94 ± 9.46	69.71
	5%	62.97 ± 11.07	84.96 ± 9.00	70.59

dCT, daily CT; MLC, multileaf collimator; MU, monitor unit.

**Figure 9:** Distribution of gamma passing rates for daily CT (dCT)-based plan and a plan with a 3% and 5% scaling in monitor units (MUs) and a 1-, 2-, and 5-mm shift in multileaf collimator (MLC) leaf (left). Dilstribution of gamma passing rates for planning CT (pCT)-based plan and a plan with a 3% and 5% scaling in MU and a 1-, 2-, and 5-mm shift in MLC leaf (right).

The ROC curves were generated for each error simulation with the EPID measurement and dCT calculated at gamma criteria of 2 mm 2%, leading to 12 curves as shown in **Figure 10**. The AUC values detected by dCT for MLC systematic shifts with 1, 2, and 5 mm are 0.63, 0.86, and 0.96, respectively. However, the AUC values for those by pCT were 0.49, 0.77, and 0.93, respectively. The ROC curves for scaling the MU were shown in **Figure 10**. The AUC values for MU scaling, using dCT-based detection, are 0.56 for the 3% offset and 0.82 for the 5% offset. For the pCT-based detection, the AUC values are 0.45 and 0.73, respectively. For MLC systematic shift, the optimal threshold of gamma passing rate was 76.80 ( ± 1 mm), 76.88 ( ± 2 mm), and 66.25 ( ± 5 mm), respectively. For MU scaling, the optimal threshold was 69.71 (3%) and 70.59 (5%).

**Figure 10:** Receiver operating characteristic (ROC) curve for a systematic shift to multileaf collimator (MLC) leaves of ±1, ± 2, and ±5 mm (left). ROC curve for scaling of the monitor unit (MU) by 3% and 5% (right).

**Figure 11** shows the case of introducing variation in dCT. The profile of introducing bias can be found easily. Nevertheless, there is no significant variation between dCT and measurement. These results indicate that using dCT as a reference is sensitive to detect bias of machine.

**Figure 11:** An example of introducing error on electronic portal image device (EPID)-based *in vivo* dosimetry during treatment.

## Discussion

The phantom results from 20 patients with different cancer sites indicated that the proposed algorithms have acceptable accuracy. The gamma passing rate for all treatment plans achieved the AAPM TG 218 report recommendations (21) (action limits: gamma passing rate ≥90%, with 3% 2 mm and a 10% dose threshold).

The correction between the results of the pCT and dCT was moderate. The coefficient of correction was approximately 0.692 (3 mm 3%), 0.684 (2 mm 3%), and 0.656 (2 mm 2%), respectively. This result reminds us that we cannot directly use pCT results and to set a threshold to replace dCT.

We also found that using dCT improved the consistency of the gamma passing rate. The standard deviations of the gamma passing rate for pCT-based were 11.52%, 14.29%, and 16.96% for 3 mm 3%, 2 mm 3%, and 2 mm 2%, respectively. The standard deviation of the gamma passing rate for dCT was 6.45%, 8.70%, and 11.94% for 3 mm 3%, 2 mm 3%, and 2 mm 2%, respectively.

This study also assesses the detectability of 2D EPID *in vivo* dosimetry for various types of variations during treatment. IGRT technology and dCT are able to reduce setup error and anatomical changes. Using the ROC methodology and different reference CT, the results show that dCT is more sensitive to variations in MLC systematic shift (AUC = 0.63–0.96) and MU scaling (AUC = 0.56–0.82).

The patient’s anatomy may have changed during the treatment course (**Figure 1**). A continuous change during the treatment course was observed for some patients in this study. **Figure 12A** presents one patient’s gamma passing rate during the first 10 days. These data were calculated on pCT. A declining trend in the pass rate was observed. For example, the gamma passing rate on day 1 for beam 140 was 83.32% (3 mm 3%), and the gamma passing rate was 38.64% (3 mm 3%) on day 10. The reason might be because of the changes in weight, respiratory motion, and random effects.

**Figure 12:** **(A)** The gamma passing rate (3 mm, 3%) between the planning CT (pCT)-based calculated dose and measured dose for a patient with 10 treatment fractions. **(B)** The gamma passing rate (3 mm, 3%) between the daily CT (dCT)-based calculated dose and measured dose for a patient.

Using dCT-based reference images will increase the gamma passing rate (**Figure 12B**). For example, the gamma passing rate of beam 140 with dCT at day 2 was 92.95% (3 mm 3%), while this passing rate was 79.03 with pCT. On day 8, we scanned the second dCT; gamma passing rate was 95.53% with dCT, pCT-based gamma passing rate was 46.96%. The average gamma passing rate increased from 75.58% to 94.93%. This finding means that patients may have anatomical changes between planning and delivery, and these anatomical changes have an impact on the transmission image pass rate. Unfortunately, considering the patient’s image dose, one patient only had one or two CT scans during treatment. Further study is required to analyze the trend of the gamma passing rate with a lower image dose.

The dCT-based 2D EPID *in vivo* dosimetry can be a choice for patient-specific QA and delivery monitoring, especially for adaptive techniques. The reliability of dCT in detecting mechanical errors is improved by separating the changes in the patient’s anatomy and setup errors. **Figures 9** and **10** show that dCT has the detectability in mechanical error. For online adaptive radiotherapy, implementing a patient-specific QA protocol with patients on the couch is difficult. Patients can undergo CT scans before delivery and dose verification during actual treatment. The whole process does not require patient movement. However, a real-time monitor may still need to be developed in the future, which can stop delivery immediately when abnormal detection is detected.

The image quality of CT may have an impact on the calculated image. Although a recent study indicated that cone beam computed tomography (CBCT) images can be used for reference image calculation (18, 28, 29), the Monte Carlo method still requires high-precision image quality. Meanwhile, the CT dose and scan time should be considered in the QA protocol design. Similar to diagnosis CT scanning, an appropriate balance was required for image quality and image dose. A prior study demonstrated that low-dose CT can reduce the radiation dose by approximately 50% compared with standard-dose CT and does not significantly affect image quality or diagnostic performance in fracture detection (30). The balance between dose and image quality should be optimized in future studies.

A proportion of fields (21%) fell into the common gamma passing rate critical area (2 mm 3%, passing rate >90%) in our results. We reviewed all patients’ dCT images, and no abnormal anatomical or position changes were observed. Direct use of 90% as the threshold may not be appropriate for transmission image comparison. Currently, there is no consensus on the criteria for patient-specific *in vivo* portal image dosimetry. Our study shows that *in vivo* dosimetry may use a different criterion from phantom QA.

In this study, only the 2D method was used and investigated. Compared to the 3D method, the main disadvantage of the 2D method is the complexity of understanding how differences in the dose at the EPID plane are related to differences in the dose to the patient (31). Combining the back-projection algorithm for 3D *in vivo* dose distribution reconstruction is another option for *in vivo* dose monitoring (32, 33). In some studies, the 3D approach showed a higher sensitivity and specificity than the 2D method (31), and the 2D approach could not combine dose-volume histogram (DVH) for analysis. However, the 2D method also has advantages in rapid detection and monitoring, which do not require data from all fields. MLC leaves systematic offsets are of excellent detectability. MU scaling offsets are of intermediate detectability. However, there is often random bias in the treatment process, which needs to be further analyzed.

There are some limitations in this study. Because of the space constraints between the couch and EPID, only fields less than 27 cm * 27 cm could be enrolled in this study. It is important to note that this study was not considered adaptive radiotherapy because the aim of this study was to integrate the QA process into the actual treatment of patients. CT scan and treatment are continuous, so it is difficult to re-segment and generate plan on dCT in our institution.

## Conclusion

This study shows the feasibility and effectiveness of the method using 2D EPID portal image and dCT-based *in vivo* dosimetry for verification of IMRT during treatment. The dCT-based *in vivo* dosimetry has better sensitivity and specificity to identify the variation of IMRT in MLC-related and dose-related errors than pCT-based.

## Data Availability Statement

The data analyzed in this study are subject to the following licenses/restrictions: These datasets can apply to EPID *in vivo* dosimetry research. Requests to access these datasets should be directed to 411593150@qq.com.

## Ethics Statement

The studies involving human participants were reviewed and approved by ethics committee, Fudan University Shanghai Cancer Center. The patients/participants provided their written informed consent to participate in this study.

## Author Contributions

BF: drafting the article. BF: processing the data, developing the deep learning model and script. BF, JW, LC, and EM: acquisition of data and generated research ideas. BF, JZ, and WH: provided guidance on methodology and overall project and reviewed the article. BF and WH: provided lab and technical support. All authors contributed to the article and approved the submitted version.

## Funding

This work is supported the Shanghai Committee of Science and Technology Fund (19DZ1930902, 21Y21900200) and Xuhui District Artificial Intelligence Medical Hospital Cooperation Project (2020-009, 2021-012).

## Conflict of Interest

The authors declare that the research was conducted in the absence of any commercial or financial relationships that could be construed as a potential conflict of interest.

## Publisher’s Note

All claims expressed in this article are solely those of the authors and do not necessarily represent those of their affiliated organizations, or those of the publisher, the editors and the reviewers. Any product that may be evaluated in this article, or claim that may be made by its manufacturer, is not guaranteed or endorsed by the publisher.
